The article "Interpretable Detection and Location of Myocardial Infarction Based on Ventricular Fusion Rule Features" was published in 2021. Journal: J Healthc Eng.

# Interpretable Detection and Location of Myocardial Infarction Based on Ventricular Fusion Rule Features

**DOI:** 10.1155/2021/4123471

**Published:** 2021-10-12

**Authors:** Wenzhi Zhang, Runchuan Li, Shengya Shen, Jinliang Yao, Yan Peng, Gang Chen, Bing Zhou, Zongmin Wang

**Affiliations:** ^1^School of Information Engineering, Zhengzhou University, Zhengzhou 450000, China; ^2^Collaborative Innovation Center for Internet Healthcare, Zhengzhou University, Zhengzhou 450000, China; ^3^Zhengzhou University of Economics and Business, Zhengzhou Henan 450000, China

## Abstract

Myocardial infarction (MI) is one of the most common cardiovascular diseases threatening human life. In order to accurately distinguish myocardial infarction and have a good interpretability, the classification method that combines rule features and ventricular activity features is proposed in this paper. Specifically, according to the clinical diagnosis rule and the pathological changes of myocardial infarction on the electrocardiogram, the local information extracted from the Q wave, ST segment, and T wave is computed as the rule feature. All samples of the QT segment are extracted as ventricular activity features. Then, in order to reduce the computational complexity of the ventricular activity features, the effects of Discrete Wavelet Transform (DWT), Principal Component Analysis (PCA), and Locality Preserving Projections (LPP) on the extracted ventricular activity features are compared. Combining rule features and ventricular activity features, all the 12 leads features are fused as the ultimate feature vector. Finally, eXtreme Gradient Boosting (XGBoost) is used to identify myocardial infarction, and the overall accuracy rate of 99.86% is obtained on the Physikalisch-Technische Bundesanstalt (PTB) database. This method has a good medical diagnosis basis while improving the accuracy, which is very important for clinical decision-making.

## 1. Introduction

MI [1] refers to a cardiovascular disease in which the coronary blood supply is drastically reduced or interrupted, causing serious and long-lasting ischemia of myocardial cells and ultimately leading to myocardial cell damage and even necrosis. Therefore, early detection and prevention of MI are of great significance, which can ensure the safety of patients' lives [2]. Myocardial enzymes usually are the main indicator for diagnosing MI. But, in the early rescue period of acute myocardial infarction, myocardial enzymes are often not elevated, and it is difficult to provide early clinical warning [3]. ECG has the advantages of celerity and low cost, so it is a common method for diagnosing MI. The electrocardiogram is a key indicator for early warning and diagnosis of MI [4, 5].

Clinicians and ECG experts recognize MI based on changes of ECG waveform and diagnosis experience. With the development of computer information technology, automatic analysis of electrocardiogram has received widespread attention. Applying computer-assisted intelligent detection to the classification of MI can help doctors diagnose MI more accurately and reduce the burden on doctors. In the current study, a variety of classification algorithms for identifying MI have been proposed, which are mainly divided into deep learning and feature engineering according to the research direction. Deep learning is classified in an end-to-end manner and has high performance, so it is widely used for MI classification. However, it does not pay attention to data processing and is dedicated to the performance of the classifier, so it cannot analyze the impact of specific features on the classification performance. The classification based on feature engineering is to analyze the ECG data, extract some useful data, or make a combination of data and perform classification according to these data. Its performance depends on the extracted features. Therefore, fully mining ECG data based on clinical medical principles not only has good interpretability but also helps to improve classification performance.

In this paper, the principal features based on the doctor's diagnosis rule [6–8] have been further calculated and applied. For the T wave and ST segment amplitude elevation or depression standard, the doctor judges whether it is elevated or depressed based on R wave and the baseline of the heartbeat; and, for abnormal Q waves, the judgment conditions are not limited to the amplitude. Therefore, doctors judge whether the patient is eligible for MI based on one or even three of the descriptions.  Figure 1 shows the different morphological features of MI.

Although these traditional features are the key to detecting myocardial infarction, in a general sense, myocardial infarction is the infarction of myocardial cells in various parts of the ventricle. Therefore, it is necessary to consider the global activity information of the ventricle. While extracting rule features, this method compares the performance of three technologies of DWT, PCA, and LPP on ventricular activity feature compression. Then the clinical rule features and the compressed ventricular activity features are fused. Finally, XGBoost is used to classify the fused features, and the tenfold cross-validation method is used for testing. The proposed method not only effectively interprets the classification basis but also makes full use of ventricular activity information, which improves the accuracy of myocardial infarction classification. The main contributions of this paper are as follows:

1. According to the clinical diagnosis significance, it not only maps the features of the doctor's diagnosis rule but also considers the information of ventricular activity. Therefore, the proposed ventricular fusion rule features demonstrate myocardial infarction information comprehensively.
2. The DWT compression method not only removes the redundant information of the ventricular activity features but also effectively retains the detailed information. Compared with PCA and LPP, it shows better performance in ventricular activity features.
3. The XGBoost model with ventricular fusion rule features is employed to classify myocardial infarction, health, and other diseases and can locate 8 types of myocardial infarction, which is very important for clinical diagnosis.

The rest of this paper is structured as follows: Section 2 briefly introduces related work.  Section 3 details the method of myocardial infarction. The experimental analysis results are introduced in Section 4.  Section 5 summarizes the full text.

## 2. Related Work

In recent years, with the development of artificial intelligence, intelligent detection of MI has become a research focus. Researchers have developed a variety of classification methods, mainly including deep learning-based methods and feature extraction-based methods.

### 2.1. Myocardial Infarction Classification Based on Deep Learning

Since there is no need to manually design feature extractors and the classification performance is significant, deep learning is widely used in myocardial infarction detection [9–16]. Acharya et al. [9] used a convolutional neural network to detect myocardial infarction. This model has high classification performance for noisy data without feature design and obtains an accuracy of 95.22%. Lui and Chow [10] used a model combining convolutional neural network and cyclic neural network to classify myocardial infarction, as well as normal and other heartbeats after heartbeat segmentation. In order to reduce the computational complexity, some methods [10, 11] only focus on single-lead classification but relatively reduce the accuracy. In deep learning, researchers strive to improve the accuracy of myocardial infarction classification through models. These methods do not require medical-related prior knowledge, and the classification accuracy is improved with big data, but because the details of the internal selection features are not clear, the ground of neural network classification cannot be known. This is a problem that cannot be ignored for medical treatment, and feature-based detection and classification methods have gradually become the focus of research.

### 2.2. Myocardial Infarction Classification Based on Feature Engineering

Feature-based classification of myocardial infarction [17–31] requires a comprehensive understanding of the data, so that the algorithm is easy to understand and interpret; and its classification accuracy usually depends on the designed features. Therefore, in order to obtain better recognition performance, some studies not only extract original physiological features but also use various techniques to extract advanced features [18–21]. Specifically, the RR interval [4], amplitude [22–24, 26], area [22, 27, 28], and other original features are extracted from the electrocardiogram. Arif et al. [22] extracted the morphological features such as the T wave amplitude, Q wave, and ST segment deviation value of the heartbeat for accurate classification, and the K-Nearest Neighbor (KNN) classifier recognized 10 types of myocardial infarction and obtained a total accuracy of 98.3%. Dohare et al. [23] extracted the amplitude, area, average, standard deviation, and other statistical features of P wave, QRS wave, and T wave as the original features and, through Principal Component Analysis dimensionality reduction processing, selected the most important 14 features for classification and finally achieved a classification accuracy of 96.66%. At present, most of the literature uses feature transformation and other techniques [29–33] to extract the advanced features of the corresponding heartbeat, such as wavelet coefficients [29, 31–33], Discrete Cosine Transform [30], and Empirical Mode Decomposition [31]. Sharma et al. [30] designed a new wavelet filter to extract the multiscale ambiguity coefficient and detail coefficient of the heartbeat and finally used KNN for myocardial infarction classification and obtained 99.62% classification accuracy. Acharya et al. [31] performed three transformations on each heartbeat of lead II and then compressed them with the LPP. Comparing the transformation effects of Discrete Cosine Transform (DCT), Discrete Wavelet Transform (DWT), and Empirical Mode Decomposition (EMD), the DCT was the best, and its accuracy was 98.5%. Acharya et al. [31] used wavelet transform to get scale coefficient features, and the KNN was employed for MI classification.

Although there is so much work in the detection of myocardial infarction [34, 35], there is still necessity for further exploration. The ECG feature that reflects the status of MI patients is not widely used, but the features composed of the amplitude and interval of the T wave, Q wave, and ST segment have achieved good results. Some of the above literatures [22–26, 36, 37] have considered these features, but the principal features based on the doctor's diagnosis rule [6–8] have not been further calculated and applied. For the T wave and ST segment amplitude elevation or depression standard, the doctor judges whether it is elevated or depressed based on the baseline of the heartbeat; and, for abnormal Q waves, the judgment conditions are not limited to the amplitude. Therefore, this work extracts not only the rule features of doctors but also the ventricular activity features which include all samples of the QT segment. Then it compares the compression effects of various techniques on ventricular activity features, the purpose of which is to remove redundant information and reduce computational complexity. Finally, the XGBoost algorithm is used to classify the features of ventricular fusion rule features, which include the ventricular activity features and the rule features. Based on the principle of myocardial infarction, this model has a high degree of recognition of the location of myocardial infarction. When myocardial infarction occurs, it can effectively help clinicians to judge and diagnose myocardial infarction in time. The relevant literatures in the related work are summarized in Table 1.

## 3. Methods

This paper mainly identifies 8 different parts of myocardial infarction, as well as health (H) and other diseases (O). These 8 parts are anterior (A), anterolateral (AL), anterior septum (AS), inferior (I), inferior lateral (IL), inferior posterior (IP), inferior posterior lateral (IPL), and posterior (P). Myocardial infarction classification usually includes three main steps: firstly, remove the baseline drift and high-frequency noise of the ECG signal, and detect the QRS complex wave and T wave according to the principle of myocardial infarction; secondly, extract rule features and ventricular activity features according to doctor's diagnosis rules and myocardial infarction pathology; finally, XGBoost algorithm is used for the classification of myocardial infarction.  Figure 2 shows the flow of myocardial infarction classification algorithm.

### 3.1. ECG Signal Preprocessing

The human body's ECG signal is weak, and noise has a great influence on the shape and details of the waveform, which often hinders the recognition of diseases. Denoising is the first step in waveform location analysis. Wavelet transform [38] is a signal time-frequency analysis method. It has the ability to characterize the local characteristics of the signal in both time and frequency domains. Therefore, it is suitable for analyzing nonstationary signals and extracting local characteristics of signals. In this paper, wavelet transform is used to remove baseline drift and high-frequency noise. The expansion of the function *f*(*t*) under the wavelet basis function *ψ*_*a*,*b*_(*t*) is continuous wavelet transform, and its definition is shown in the following formula:

(1) $$\begin{array}{c} W_{f}\left(a,b\right)=\langle f\left(t\right)\cdot \psi_{a,b}\left(t\right)\rangle =\frac{1}{\sqrt{a}}\int_{-\infty }^{+\infty }f\left(t\right)\psi \left(\frac{t-b}{a}\right)dt, \end{array}$$

where *a* is the scale factor and *b* is the transformation factor; through these two parameters, the wavelet function can be stretched along the time axis and the wavelet coefficients can be calculated until the end of the signal.

The essence of denoising is to decompose the different frequency parts of the signal into different scale spaces and then remove the wavelet coefficients on the corresponding scale of the noise and retain the wavelet coefficients obtained from the useful signal; finally, the signal is reconstructed. Figures 3 and 4 show the ECG data before and after denoising.

For waveform segmentation, the signal is wavelet decomposed by the Mexican hat basis function to separate the QRS complex wave [39] in this paper. This technology decomposes signals of different frequencies into different scales, distinguishing QRS complex waves. After detecting the QRS complex, the search window of the P wave and T wave is defined according to the calculated RR interval and relative to the position of the QRS complex. In order to verify the accuracy of the extracted features, this paper verifies on private dataset. The collaborative center ECG data is our private data which is a 12-lead ECG data record. The subjects were men aged between 21 and 91 years and women aged between 29 and 89 years. 128 samples/sec are recorded for each lead for digitization. Then each record is resampled to 360 samples/sec. The signal voltage is within 5 mV with 8-bit resolution. The doctor randomly selects clearer data from the collected 24-hour Holter ECG records for labeling, one hour during the day and one hour at night. Each piece of data has approximately 1.3 million sampling points. The test results are shown in Table 2. The detection is shown in Figure 5.

### 3.2. Feature Extraction

When myocardial infarction occurs, the abnormal wave pattern continues to change over time. In the early stage of myocardial infarction, the T wave and ST segment are elevated at the same time; after the myocardial infarction lasts for a few hours, the ST segment arch is elevated, forming a one-way curve, abnormal Q waves appear, and the T wave is gradually inverted. In the subacute phase, the ST segment returns to the baseline I point, the T wave gradually becomes flat, and the abnormal Q wave persists; in the old phase, the ST segment and T wave return to normal, but the abnormal Q wave persists. ST segment, T wave, and Q wave have different morphological criteria due to different leads. Therefore, it is not possible to simply extract the amplitude or duration of the band nor only describe the information of one band. It is necessary to associate multiple waveforms for a comprehensive description. Based on the research of related literature [6–8] combined with doctor's diagnosis rules, this paper extracts the following myocardial infarction-related feature groups.  Figure 6 is the annotation of extracted features. Among them, ST segment, T wave, and Q wave are the ground for doctors to diagnose myocardial infarction, so they are integrated as rule features, and the specifics are shown in formulas (2)–(8). The specific calculation formula for ventricular activity features is formula (9).  Table 3 summarizes the features' descriptions extracted in this paper:

(a) ST segment features description: these features include the amplitude difference between the *J* point (QRS end point) and the baseline (QRS starting point) and the amplitude difference between the T wave start point and the *J* point. When myocardial infarction occurs, the ST segment is abnormally elevated or depressed, and the doctor judges whether the ST segment is elevated or depressed based on the magnitude of the amplitude difference.
  (2) $$\begin{array}{c} J_{\_}\mathrm{relative}=J_{\_}\mathrm{amp}-I_{\_}\mathrm{amp,} \end{array}$$
  (3) $$\begin{array}{c} ST_{\_}\mathrm{relative}=\mathrm{Tstar}t_{\_}\mathrm{amp}-J_{\_}\mathrm{amp}. \end{array}$$
(b) Q wave features description: these features include the duration of the Q wave and the ratio of the amplitude of the Q wave to the R wave. When the myocardial infarction progresses to the later stage, abnormal Q waves will appear. Its specific features are that the Q wave is broadened, and the amplitude exceeds a certain proportion of the R wave in the same lead.
  (4) $$\begin{array}{c} Q_{\_}\mathrm{ratio}=\left|\frac{Q_{\_}\mathrm{amp}-I_{\_}\mathrm{amp}}{R_{\_}\mathrm{amp}-I_{\_}\mathrm{amp}}\right|=\left|\frac{Q_{\_}\mathrm{relative}}{R_{\_}\mathrm{relative}}\right|, \end{array}$$
  (5) $$\begin{array}{c} Q_{\_}\mathrm{interval}=\frac{Q_{\_}\mathrm{pos}-I_{\_}\mathrm{pos}}{\text{SR}}. \end{array}$$
(c) T wave features description: these features include the ratio of the amplitude of the T wave to the R wave, the amplitude difference between the T wave and its start point, and the amplitude difference between the T wave and its end point. Different leads have different T wave morphology standards. To determine the T wave morphology change needs to be based on the R wave amplitude or the amplitude of the start and end points of the T wave. When the T wave is higher than a certain proportion of the R wave, it is usually a towering T wave, and when the T wave is lower than a certain proportion of the R wave or the relative starting point of the T wave is lower than a certain amplitude, it is low and flat. The difference in amplitude between the T wave and its start and end points describes whether the T wave is inverted or upright.
  (6) $$\begin{array}{c} T_{\_}\mathrm{ratio}=\frac{T_{\_}\mathrm{amp}-I_{\_}\mathrm{amp}}{R_{\_}\mathrm{amp}-I_{\_}\mathrm{amp}}=\frac{T_{\_}\mathrm{relative}}{R_{\_}\mathrm{relative}}, \end{array}$$
  (7) $$\begin{array}{c} \mathrm{Tstar}t_{\_}\mathrm{relative}=T_{\_}\mathrm{amp}-\mathrm{Tstar}t_{\_}\mathrm{amp,} \end{array}$$
  (8) $$\begin{array}{c} \mathrm{Ten}d_{\_}\mathrm{relative}=T_{\_}\mathrm{amp}-\mathrm{Ten}d_{\_}\mathrm{amp}. \end{array}$$
(d) QT segment features description: the QT segment is the ECG record from the beginning of the Q wave to the end of the T wave, including QRS complex wave and ST-T segment. Since the QRS wave represents the time of ventricular depolarization and the ST-T wave represents the time of slow ventricular repolarization, the QT segment is a total measurement of ventricular activity. Myocardial infarction generally occurs in the ventricle, so the record of ventricular activity has a more comprehensive and accurate description of myocardial infarction. In this paper, QT segments are extracted and unified to 1000 samples as ventricular activity feature.
  (9) $$\begin{array}{c} QT=\left\{x_{1_{\_}}\text{amp},x_{2_{\_}}\text{amp}\ldots x_{m_{\_}}\text{amp}\right\}\;m\text{Î}\left[I,\text{Tend}\right]. \end{array}$$

### 3.3. Feature Compression

In this paper, considering that myocardial infarction is not simply embodied in a fixed feature, as it is a comprehensive measurement of Q wave and ST-T segment, the rule feature group is a feature map for doctors to diagnose myocardial infarction, which is not needed feature compression in this work. For the ventricular activity features, all sampling points of the QT segment are included. Simply extracting all samples is often mixed with redundant information, and the feature dimension is too high to make the calculation complicated, so it needs to be compressed. Different feature compression methods have different effects on the same data. Therefore, for the ventricular activity features, this paper used three techniques for comparison: DWT, PCA, and LPP. The 1000 samples of ventricular activity features are compressed into 32 features.

#### 3.3.1. Discrete Wavelet Transform

Discrete Wavelet Transform is a time domain-frequency domain transform analysis method [40], which decomposes the signal into different frequency components through high-pass filtering and low-pass filtering. The output of the high-pass filter is the detail coefficient, which represents the high-frequency information of the signal; the output of the low-pass filter is the approximate coefficient, which represents the low-frequency information of the signal. In this work, db4 wavelet is used to decompose the feature of ventricular activity in five levels. After the ECG signal is processed by the db4 wavelet function, the coefficients are smoother, and at the same time it is guaranteed to be closer to the original waveform. Discrete Wavelet Transform is to sample the scale and translation parameters of the continuous wavelet in the above formula (1), which is defined as follows:

(10) $$\begin{array}{c} W\left(a,b\right)=\frac{1}{\sqrt{a}}\sum_{R}f\left(n\right)\psi_{a,b}\left(n\right). \end{array}$$

#### 3.3.2. Principal Component Analysis

Principal Component Analysis is a dimensionality reduction method based on orthogonal transformation [41], which recombines relevant indicators into irrelevant comprehensive indicators. This technology uses linear projection to map high-dimensional data to low-dimensional space while ensuring that the variance of the projected data is maximized. In this work, considering that the ECG data bands and adjacent lead data are generally correlated, resulting in greater redundancy, the global key features are extracted. The principal formula of Principal Component Analysis is shown as follows:

(11) $$\begin{array}{c} X_{m*k}^{\prime }=X_{m*n}V_{n*k}^{T}. \end{array}$$

When the sample is an *m* ^*∗*^ *n* matrix *X*, find the *k* ^*∗*^ *n* matrix *V*^*T*^ composed of the largest *k* eigenvectors of the matrix *X*^*T*^*X* through Singular Value Decomposition (SVD). Matrix *V*^*T*^ compresses the features of *m* columns to *k* columns.

#### 3.3.3. Locality-Preserving Projections

Local Preserving Projections are a linear dimensionality reduction technique, which reduces the spatial dimension while maintaining the internal fixed local structure [42]. After constructing an adjacency matrix representing the near-distance relationship between samples, this technology introduces the Laplace-Beltrami function and calculates the best linear approximation to obtain a locally preserved projection. This work considers that ventricular activity features of the same structure are similar, and extracting the commonality of these neighboring features can effectively compare the features. The loss function of the principle of Local Preserving Projections is shown in the following formula:

(12) $$\begin{array}{c} \sum_{ij}{\left(y_{i}-y_{j}\right)}^{2}W_{ij}. \end{array}$$

Here, *y*_*i*_ represents any data point *i* after dimensionality reduction, *y*_*j*_ represents any data point that does not contain *i* point after dimensionality reduction, and *W*_*ij*_ represents a matrix composed of the distance weight coefficients between *i* and *j* in the original space.

### 3.4. XGBoost Model Description

XGBoost is an improved algorithm based on Gradient Boosting Decision Tree (GBDT); similar to GBDT, it is an ensemble algorithm composed of multiple decision trees [43]. The basic idea is to establish K decision trees so that the predicted value of the tree group is as close as possible to the true value (accuracy) and has the greatest possible generalization ability. The structure of the algorithm is shown in Figure 7. The algorithm uses multiple iterations; each iteration produces a weak classifier, and each classifier is trained on the basis of the residual of the previous round of classifiers. Finally, the accuracy of the final classifier is continuously improved by reducing the deviation.

For the input sample *X*, the output prediction model is

(13) $$\begin{array}{c} {\hat{y}}_{i}=\sum_{k=1}^{K}f_{k}\left(x_{i}\right), \end{array}$$

where *K* is the total number of numbers, *f*_*k*_ represents the *k*-th tree, and ${\hat{y}}_{i}$ represents the prediction result of sample *x*_*i*_.

The loss function is expressed as

(14) $$\begin{array}{c} \text{Obj}\left(\theta \right)=\sum_{i=1}^{n}l\left(y_{i},{\hat{y}}_{i}\right)+\sum_{k=1}^{K}\Omega \left(f_{k}\right). \end{array}$$

Here, $l\left(y_{i},{\hat{y}}_{i}\right)$ is the training error of the sample, and Ω(*f*_*k*_)represents the regular term of the *k*-th tree. The formula is as shown in (15): *T*is the number of leaf nodes of the tree, and *w* is the output score of the leaf nodes of each tree.

(15) $$\begin{array}{c} \Omega \left(f_{t}\right)=\gamma T+\frac{1}{2}\lambda \sum_{j=1}^{T}w_{j}^{2}. \end{array}$$

Since *f* is a decision tree, not a numerical vector, it cannot directly optimize the loss function, so it is necessary to find a local optimal solution through a greedy algorithm; and the predicted score for the *t*-th tree can be expressed as

(16) $$\begin{array}{c} {\hat{y}}_{i}^{\left(t\right)}={\hat{y}}_{i}^{\left(t-1\right)}+f_{t}\left(x_{i}\right). \end{array}$$

The optimized loss function obtained by Taylor expansion formula is shown in (17), where *g*_*i*_ is the first-order derivative and *h*_*i*_ denotes the second-order derivative:

(17) $$\begin{array}{c} \mathrm{Ob}j^{t}\left(\theta \right)=\sum_{j=1}^{T}\left[g_{i}f_{t}\left(x_{i}\right)+\frac{1}{2}h_{i}f_{t}^{2}\left(x_{i}\right)\right]+\gamma T+\frac{1}{2}\lambda \sum_{j=1}^{T}w_{j}^{2}\\ =\sum_{j=1}^{T}\left[\left(\sum_{i\in I_{j}}g_{i}\right)w_{j}+\frac{1}{2}\left(\sum_{i\in I_{j}}h_{i}+\lambda \right)w_{j}^{2}\right]+\gamma T. \end{array}$$

Here, by making *G*_*j*_=∑_*i*∈*I*_*j*__*g*_*i*_ and *H*_*j*_=∑_*i*∈*I*_*j*__*h*_*i*_, the loss function can be further compressed to obtain formula (18), where the partial derivative of *w*_*j*_ can be replaced by *G*_*j*_ and *H*_*j*_. Formula (19) is obtained, and the final loss function is shown in formula (20).

(18) $$\begin{array}{c} \mathrm{Ob}j^{t}\left(\theta \right)=\sum_{j=1}^{T}\left[G_{j}w_{j}+\frac{1}{2}\left(H_{j}+\lambda \right)w_{j}^{2}\right]+\gamma T, \end{array}$$

(19) $$\begin{array}{c} w_{j}^{*}=-\frac{G_{j}}{H_{j}+\lambda }, \end{array}$$

(20) $$\begin{array}{c} \mathrm{Ob}j^{*}=-\frac{1}{2}\sum_{j=1}^{T}\frac{G_{j}}{H_{j}+\lambda }+\gamma T. \end{array}$$

The advantage of XGBoost is that it has a reliable objective function. XGBoost adds a regularization term to the objective function to make the trained model simpler and prevent overfitting. Compared with GBDT, XGBoost expands the objective function Taylor to the second order, retaining more information about the objective function, making the algorithm converge to the global optimum faster. XGBoost performs column sampling in a similar manner to random forests, which can not only reduce overfitting but also reduce calculations. In this paper, comparing the performance of multiple classifiers while considering the characteristics of the classifiers, a decision tree is selected as the base classifier. Then ensemble learning is used to alleviate data imbalance and improve classifier performance.

## 4. Results

In this part, the process and results of the experiment will be described in detail. The subject focuses on feature extraction and classification of myocardial infarction. According to clinical medical diagnosis rules and medical significance, 7 rule features are extracted and calculated as feature groups, and all samples of QT segment are extracted as ventricular activity features. In order to reduce the redundant information of the ECG data of the 12-lead ventricle and improve the efficiency of the model, three technologies of DWT, PCA, and LPP are used to transform and compare the ventricular activity features, and 32 features are obtained, respectively. Finally, the performances of the ventricular activity features with the best compression effect and the rule features and their combination on the classification effect are compared. This paper uses the PTB database. The focus is on the analysis and classification of 8 kinds of myocardial infarction, as well as health and other diseases data. A total of 37,359 heart beats were extracted, and the 10-fold cross-validation method was used for model [44]. This process divides the training set into ten subsets. For each subset, the remaining dataset is used to train the model, and then the subset is used to predict the result. This process is repeated ten times. The average of the prediction results is taken as the final prediction result. The classification results help doctors make preliminary judgments.

### 4.1. Experimental Data

The data used in this paper comes from the PTB diagnostic ECG database [45]. The PTB diagnostic ECG database includes 549 records of 290 MI, other diseases, and healthy control patients. 1 to 5 records are collected for each subject. Each record is about 2 minutes, including 15 simultaneous measurement signals: traditional 12-lead and 3 Frank-lead ECG signals. The data is shown in Table 4. In this study, a 12-lead electrocardiogram was used to analyze and classify data on 8 types of myocardial infarction, health, and other diseases.

This work classifies myocardial infarction from health (H) and other diseases (O) while classifying anterior (A), anterolateral (AL), anterior septum (AS), inferior (I), inferior lateral (IL), inferior posterior (IP), inferior posterior lateral (IPL) and posterior (P) myocardial infarctions. The extracted data is shown in Table 5.

### 4.2. Evaluation Indicator

In this paper, the experimental results are obtained by comparing the difference between the label output of the model and the real label. The evaluation indicator is based on the literature [46] using sensitivity, specificity, positive predictability, and accuracy to evaluate the results of the experiment. Sensitivity (Se) is the proportion of samples judged to be positive in all positive cases. Specificity (Sp) is the proportion of samples judged to be negative among all negative cases. The positive predictive value (+*p*) is also known as precision, which is the correct proportion of all samples that are judged to be positive. Accuracy (Acc) is the proportion of correctly classified samples to the total sample. The calculation formulas ((21)–(24)) of the four evaluation indicators are as follows:

(21) $$\begin{array}{c} \mathrm{Se}=\frac{\mathrm{TP}}{\left(\mathrm{TP+FN}\right)}, \end{array}$$

(22) $$\begin{array}{c} \mathrm{Sp}=\frac{\mathrm{TN}}{\left(\mathrm{TN+FP}\right)}, \end{array}$$

(23) $$\begin{array}{c} +p=\frac{\mathrm{TP}}{\left(\mathrm{TP+FP}\right)}, \end{array}$$

(24) $$\begin{array}{c} \mathrm{Acc}=\frac{\left(\mathrm{TP+TN}\right)}{\left(\mathrm{TP+TN+FP+FN}\right)}. \end{array}$$

### 4.3. Experiment and Result Analysis

In order to verify the effectiveness of the extracted features and compare the performances between XGBoost and other classifiers, this work conducted four sets of experiment. Experiment 1 applies three technologies to compare the ventricular activity features and verifies the effect through the XGBoost. Experiment 2 compares the performance of the rule features, the ventricular activity features, and the ventricular fusion rule features on the XGBoost. In order to verify the effectiveness of the XGBoost, Experiment 3 compares the performance of XGBoost with traditional basic classifiers. At the same time, because XGBoost belongs to ensemble learning, Experiment 4 compares it with other ensemble classifiers. Finally, the proposed method is compared with other literature methods.

#### 4.3.1. Comparative Analysis of Different Dimensionality Reduction Methods

In order to fully explore the medical significance of ECG signals in myocardial infarction, this paper extracts a total of 1000 samples of QT segment as ventricular activity features. At the same time, in order to remove the redundant information of the ventricular activity features, Experiment 1 used three different technologies of DWT, PCA, and LPP to compare the ventricular activity features.  Table 6 shows the compression effects of the three transformation techniques on ventricular activity features.

According to the experimental results, although PCA has good performance on individual classifiers, for example, reaching 93.02% on XGBoost, it does not work well on most classifiers. This is because PCA is sensitive to local singular features in the transformation process but ignores key detailed features, so the classification accuracy is relatively low. LPP has high performance on most classifiers; it reached an accuracy of more than 90% on most of them. But, for a few classifiers, the performance is poor, so the overall effect on all the classifiers is not good. DWT has achieved good performance on all classifiers, with an average classification accuracy of 90.31%. This is because DWT reduces the feature dimension while making it as close to the original signal waveform as possible, retaining the global key features, so the overall classification accuracy is higher, and it reaches 99.70% on XGBoost. Based on the above experimental results, this article will select the ventricular activity features after DWT transformation as further experiments.

#### 4.3.2. Comparative Analysis of Different Features

In order to understand and make full use of the global features of myocardial infarction, we compare and analyze the performance differences of the rule features, ventricular activity features, and ventricular fusion rule features and use the overall accuracy as the final indicator of comparison. Experiment 2 compares the performance differences of the three feature sets through XGBoost.  Table 7 shows the classification performance of three feature sets on XGBoost.

The results show that the model based on rule features has high classification performance, and its total accuracy is 99.67%. This shows that the doctor's diagnosis rules have a good effect on the recognition of myocardial infarction, and it can be classified as a strong feature by itself. The classification of myocardial infarction based on the ventricular activity features has significant performance, with an accuracy of up to 99.70%. Because it contains more heart activity information, it has improved rule features, but the improvement is not obvious. The ventricular fusion rule features use the correlation information between different segments and the global ventricular activity information, and its final classification accuracy is 99.86%. Compared with the rule features, the ventricular fusion rule feature supplements the specific details of the internal information; and, compared with the ventricular activity features, the ventricular fusion rule features add the correlation information between the segments. Therefore, compared with the other two features, the classification performance of the ventricular fusion rule feature has a certain improvement. Tables 8 and 9 and Figure 8 show the detailed classification results of the ventricular fusion rule features.

#### 4.3.3. Comparative Analysis of XGBoost and Base Classifiers

Experiment 3 compares the performance between XGBoost and traditional classifiers. This paper selects 6 basic classifiers for comparison: K-Nearest Neighbor (KNN), Gaussian Naive Bayes (GNB), Linear Discriminant Analysis (LDA), decision tree (DT), Support Vector Machine (SVM), and Logistic Regression (LR). The comparison results are shown in Table 10.

The results show that, compared to the basic classifier, XGBoost has significant performance on all three feature sets. Among them, for all classifiers, the ventricular fusion rule feature has a certain improvement in performance compared with other features. In addition to XGBoost, DT, SVM, and KNN all have good classification performance, with a classification accuracy of about 90%, but the performance of SVM is greatly affected by the feature dimension, and the classification performance is not stable.

#### 4.3.4. Comparative Analysis of Different Ensemble Methods

Experiment 4 compares the performance of XGBoost classifiers with other ensemble methods. This paper selects several common ensemble methods for comparison, such as AdaBoost, GBDT, Bagging, Random Forest, and ExtraTrees. The results are shown in Table 11.

The results show that each ensemble classifier has higher performance in each feature set. Among them, Random Forest, ExtraTrees, and XGBoost are the most prominent, achieving 99% accuracy on all feature sets. However, in a comprehensive comparison, XGBoost has the best performance, which achieves 99.6% on all feature sets, and the accuracy of ventricular fusion rule features is even 99.86%.

#### 4.3.5. Comparative Analysis with Other Studies

In order to verify the performance of the proposed method, this paper performs a comparison with other literature methods. The results are shown in Table 12. The above four experiments show that the XGBoost model based on ventricular fusion rules has better performance than the other methods in this paper, and the overall accuracy reaches 99.86%. This method can not only identify myocardial infarction, health, and other diseases but also detect 8 parts of myocardial infarction. Compared with literature [5, 28, 29, 47], the proposed method has superior results in detection and location, and it is also competitive compared to deep learning networks. Therefore, compared with the above literature results, the proposed method has excellent performance in the recognition of myocardial infarction.

## 5. Conclusion

Accurate identification of myocardial infarction based on medical principles is very important for the treatment of patients. Therefore, a classification method of myocardial infarction based on the ventricular fusion rule features and the XGBoost algorithm is proposed this paper. In the preprocessing, wavelet transform is used for denoising and waveform segmentation. Then, rule features based on clinical diagnosis rules and ventricular activity features based on myocardial infarction pathology are extracted. By comparing the compression performances of PCA, LPP, and DWT, low-dimensional and efficient ventricular activity features can be obtained. The features obtained by the above methods are fused into the final feature group as ventricular fusion features. For MI classification, compared with other algorithms combined with 10-fold cross-validation, the classification method based on the XGBoost algorithm obtained a total accuracy of 99.86%. The main advantages of the proposed method include the following: fully consider the development process of myocardial infarction to extract comprehensive feature information; compare multiple compression methods and classification strategies to get the best myocardial infarction detection and location strategy; the ventricular fusion rule features extracted based on the ECG specific waveform changes of myocardial infarction and the doctor's diagnosis strategy show more vital clinical significance and excellent results.

However, the rule features proposed in this paper do not describe the doctor's diagnosis rule comprehensively, such as the internal changes of ST segment. In the future, more interpretability and simplified features based on clinical diagnosis rules are applied to the detection and location of myocardial infarction. Meanwhile, the above methods still rely on a mass of clinical ECG data, so we will focus on the collection and processing of ECG data.

## Figures and Tables

**Figure 1:** Different forms of myocardial infarction. (a) The morphology is manifested as only abnormal Q waves. (b) The morphological manifestation is ST segment elevation and T wave height. (c) The morphology is ST segment elevation, T wave inversion, and normal Q wave. (d) The appearance of abnormal Q wave and T wave inversion.

**Figure 2:** Myocardial infarction classification algorithm flow.

**Figure 3:** Raw data of myocardial infarction.

**Figure 4:** Myocardial infarction data after denoising.

**Figure 5:** Position mark of each waveform detected.

**Figure 6:** The annotation of extracted features.

**Figure 7:** XGBoost algorithm structure.

**Figure 8:** Confusion matrix based on classification results of XGBoost with ventricular fusion rule features.

**Table 1:** Summary of related work.

Method	Feature	Literatures
Deep learning	End-to-end	[9–16]

Machine learning	Morphology	[22–26, 36, 37]
	Interval	[4, 25]
	Area	[22, 27, 28]
	Wavelet coefficients	[18, 20, 21, 25, 29, 31–33]
	Discrete Cosine Transform	[30]
	Empirical Mode Decomposition	[31]

**Table 2:** Statistical results of wave detection in collaborative center ECG data.

Records	R wave			P wave			T wave		
	+*p*%	Se%	Acc%	+*p*%	Se%	Acc%	+*p*%	Se%	Acc%
001	99.78	100	99.78	99.93	99.95	99.89	99.79	99.87	99.67
002	99.94	100	99.94	99.92	99.92	99.84	99.79	99.87	99.67
003	99.93	99.93	99.87	99.84	99.96	99.81	99.93	99.90	99.84
004	99.89	100	99.89	99.86	99.86	99.73	99.76	99.83	99.59
005	99.91	100	99.91	99.88	100	99.88	99.95	100	99.95

**Table 3:** ECG signal features in this paper.

Number	ECG signal features	Introduction of ECG signal feature parameters
1	Rule features	Including ST segment features description, Q wave features description, and T wave features description, a total of 7 features

2	Ventricular activity features	Including 1000 sample points of the QT segment

3	Ventricular fusion rule features	Combining ruler features and ventricular activity features

**Table 4:** PTB dataset diseases.

No.	Diagnostic class	Records
1	Bundle branch block	17
2	Cardiomyopathy	17
3	Dysrhythmia	16
4	Healthy control	80
5	Heart failure	3
6	Myocardial hypertrophy	7
7	Myocardial infarction	368
8	Myocarditis	4
9	N/A: clinical summary not available	27
10	Palpitation	1
11	Stable angina	2
12	Unstable angina	1
13	Valvular heart disease	6

**Table 5:** Total number of heart beats extracted.

Class	Number of beats
A	5001
AL	4695
AS	3219
I	5395
IL	3391
IP	503
IPL	1739
P	460
H	5820
O	7136
Total	37359

**Table 6:** Performance comparison of each classifier on PCA, LPP, and DWT.

Classifier	PCA (%)	LPP (%)	DWT (%)
KNN	53.94	97.74	98.15
GNB	26.70	23.43	48.00
LDA	13.88	27.07	76.00
LR	14.31	39.75	82.17
DT	73.16	98.71	92.84
SVM	61.17	37.10	98.55
Random forest	80.75	99.43	99.46
AdaBoost	73.80	98.31	92.46
ExtraTrees	70.80	99.19	99.59
Bagging	88.12	99.19	98.89
GBDT	67.98	99.65	97.96
*XGBoost*	93.02	99.65	99.70
*Average*	59.80	76.60	90.31

**Table 7:** Classification performance of three feature sets on XGBoost.

Classifier	Rule features (%)	Ventricular activity features (%)	Ventricular fusion rule features (%)
XGBoost	99.67	99.70	99.86

**Table 8:** XGBoost with ventricular fusion rule features of classification results specific category statistics.

	A	AS	AL	I	IL	IP	IPL	P	H	O
A	500	0	0	0	0	0	0	0	0	0
AS	1	468	0	0	0	0	0	0	0	0
AL	0	0	320	0	0	0	0	1	0	0
I	0	0	0	537	1	0	0	0	0	1
IL	0	0	0	0	339	0	0	0	0	0
IP	0	0	0	0	0	50	0	0	0	0
IPL	0	0	0	0	0	0	173	0	0	0
P	0	0	0	0	0	0	0	46	0	0
H	0	0	0	0	0	0	0	0	582	0
O	0	0	0	0	0	0	0	0	1	710

**Table 9:** XGBoost with ventricular fusion rule features of classification results.

	TP	TN	FP	FN	Se	Sp	+*p*	Acc
A	500	3229	1	0	100	99.97	99.80	99.97
AS	468	3261	0	1	99.79	100	100	99.97
AL	320	3409	0	1	99.69	100	100	99.97
I	537	3191	0	2	99.63	100	100	99.95
IL	339	3390	1	0	100	99.97	99.71	99.97
IP	50	3680	0	0	100	100	100	100
IPL	173	3557	0	0	100	100	100	100
P	46	3683	1	0	100	99.97	97.87	99.97
H	582	3147	1	0	100	99.97	99.83	99.97
O	710	3019	1	1	99.86	99.97	99.86	99.95

**Table 10:** Detailed performance comparison between XGBoost and other basic classifiers.

Classifier	Rule features (%)	Ventricular activity features (%)	Ventricular fusion rule features (%)
GNB	42.68	48.00	56.11
LDA	55.63	76.00	84.98
LR	61.98	82.17	92.57
DT	93.53	92.84	95.65
SVM	89.00	98.55	99.08
KNN	95.33	98.15	99.06
*XGBoost*	99.67	99.70	99.86

**Table 11:** Detailed performance comparison between XGBoost and other ensemble classifiers.

Classifier	Rule features (%)	Ventricular activity features (%)	Ventricular fusion rule features (%)
Random Forest	99.27	99.46	99.75
ExtraTrees	99.51	99.59	99.75
AdaBoost	94.45	92.46	95.54
Bagging	98.25	97.98	98.60
GBDT	98.04	97.96	99.19
*XGBoost*	99.67	99.70	99.86

**Table 12:** Comparison of the proposed method with other related literature.

Reference	Class number	Feature	Classifier	Performance (%)
Lin et al. [5]	2	MODWPT, statistical	KNN	Acc = 99.57; Se = 99.82; Sp = 98.79
Baloglu et al. [12]	11	End-to-end	CNN	Acc = 99.78;
Han and Shi [13]	7	End-to-end	ResNet	Acc = 99.72; Se = 99.63; Sp = 99.72;
Han and Shi [28]	2	MODWPT, morphological	SVM	Acc = 99.81; Se = 99.56; +*p* = 99.74
Acharya et al. [29]	11	DWT	KNN	Acc = 98.80; Se = 99.45; Sp = 96.27
Padhy and Dandapat [47]	6	Singular Value Decomposition	SVM	Acc = 95.30; Se = 94.60; Sp = 96.00
Liu et al. [48]	6	End-to-end	CNN	Acc = 99.81
*Proposed*	10	DWT, rule features	XGBoost	Acc = 99.86; Se = 99.86; Sp = 99.86

## Data Availability

All the datasets used to support the findings of this study are included within the article. All datasets used to support the findings of this study were supplied by the publicly available PTB database from the Massachusetts Institute of Technology. The URL to access this data is https://www.physionet.org/cgi-bin/atm/ATM. The coding and source code used to support the findings of this study have not been made available because the source code in this article is part of a national project and is a trade secret.

## References

[1] Miranda D. F., Lobo A. S., Walsh B., Sandoval Y., Smith S. W. (2018). New insights into the use of the 12-lead electrocardiogram for diagnosing acute myocardial infarction in the emergency department. *Canadian Journal of Cardiology*.

[2] Boersma E., Maas A. C., Deckers J. W., Simoons M. L. (1996). Early thrombolytic treatment in acute myocardial infarction: reappraisal of the golden hour. *The Lancet*.

[3] Sobel B. E., Shell W. E. (1972). Serum enzyme determinations in the diagnosis and assessment of myocardial infarction. *Circulation*.

[4] Kayikcioglu İ., Akdeniz F., Köse C., Kayikcioglu T. (2020). Time-frequency approach to ECG classification of myocardial infarction. *Computers & Electrical Engineering*.

[5] Lin Z., Gao Y., Chen Y., Ge Q., Mahara G., Zhang J. (2020). Automated detection of myocardial infarction using robust features extracted from 12-lead ECG. *Signal, Image and Video Processing*.

[6] Zimetbaum P. J., Josephson M. E. (2003). Use of the electrocardiogram in acute myocardial infarction. *New England Journal of Medicine*.

[7] Thygesen K., Alpert J. S., White H. D. (2007). Universal definition of myocardial infarction. *Journal of the American College of Cardiology*.

[8] Goldberger A. L., Goldberger Z. D., Shvilkin A. (2017). *Clinical Electrocardiography: A Simplified Approach E-Book*.

[9] Acharya U. R., Fujita H., Oh S. L., Hagiwara Y., Tan J. H., Adam M. (2017). Application of deep convolutional neural network for automated detection of myocardial infarction using ECG signals. *Information Sciences*.

[10] Lui H. W., Chow K. L. (2018). Multiclass classification of myocardial infarction with convolutional and recurrent neural networks for portable ECG devices. *Informatics in Medicine Unlocked*.

[11] Kora P. (2017). ECG based myocardial infarction detection using hybrid firefly algorithm. *Computer Methods and Programs in Biomedicine*.

[12] Baloglu U. B., Talo M., Yildirim O., Tan R. S., Acharya U. R. (2019). Classification of myocardial infarction with multi-lead ECG signals and deep CNN. *Pattern Recognition Letters*.

[13] Han C., Shi L. (2020). ML-ResNet: a novel network to detect and locate myocardial infarction using 12 leads ECG. *Computer Methods and Programs in Biomedicine*.

[14] Hao P., Gao X., Li Z., Zhang J., Wu F., Bai C. (2020). Multi-branch fusion network for myocardial infarction screening from 12-lead ECG images. *Computer Methods and Programs in Biomedicine*.

[15] Prabhakararao E., Dandapat S. (2020). Myocardial infarction severity stages classification from ecg signals using attentional recurrent neural network. *IEEE Sensors Journal*.

[16] Sugimoto K., Kon Y., Lee S., Okada Y. (2019). Detection and localization of myocardial infarction based on a convolutional autoencoder. *Knowledge-Based Systems*.

[17] Sharma L. D., Sunkaria R. K. (2020). Myocardial infarction detection and localization using optimal features based lead specific approach. *IRBM*.

[18] Sridhar C., Lih O. S., Jahmunah V. (2020). Accurate detection of myocardial infarction using non linear features with ECG signals. *Journal of Ambient Intelligence and Humanized Computing*.

[19] Heo J., Lee J. J., Kwon S., Kim B., Hwang S. O., Yoon Y. R. (2020). A novel method for detecting ST segment elevation myocardial infarction on a 12-lead electrocardiogram with a three-dimensional display. *Biomedical Signal Processing and Control*.

[20] Liu J., Zhang C., Zhu Y., Ristaniemi T., Parviainen T., Cong F. (2020). Automated detection and localization system of myocardial infarction in single-beat ECG using Dual-Q TQWT and wavelet packet tensor decomposition. *Computer Methods and Programs in Biomedicine*.

[21] Choudhary P. S., Dandapat S. An evaluation of machine learning classifiers for detection of myocardial infarction using wavelet entropy and eigenspace features.

[22] Arif M., Malagore I. A., Afsar F. A. (2012). Detection and localization of myocardial infarction using k-nearest neighbor classifier. *Journal of Medical Systems*.

[23] Dohare A. K., Kumar V., Kumar R. (2018). Detection of myocardial infarction in 12 lead ECG using support vector machine. *Applied Soft Computing*.

[24] Remya R. S., Indiradevi K. P., Babu K. K. A. (2016). Classification of myocardial infarction using multi resolution wavelet analysis of ECG. *Procedia Technology*.

[25] Diker A., Cömert Z., Avci E., Velappan S. Intelligent system based on genetic algorithm and support vector machine for detection of myocardial infarction from ECG signals.

[26] Sun L., Lu Y., Yang K., Li S. (2012). ECG analysis using multiple instance learning for myocardial infarction detection. *IEEE Transactions on Biomedical Engineering*.

[27] Safdarian N., Dabanloo N. J., Attarodi G. (2014). A new pattern recognition method for detection and localization of myocardial infarction using T-wave integral and total integral as extracted features from one cycle of ECG signal. *Journal of Biomedical Science and Engineering*.

[28] Han C., Shi L. (2019). Automated interpretable detection of myocardial infarction fusing energy entropy and morphological features. *Computer Methods and Programs in Biomedicine*.

[29] Acharya U. R., Fujita H., Sudarshan V. K. (2016). Automated detection and localization of myocardial infarction using electrocardiogram: a comparative study of different leads. *Knowledge-Based Systems*.

[30] Sharma M., Tan R. S., Acharya U. R. (2018). A novel automated diagnostic system for classification of myocardial infarction ECG signals using an optimal biorthogonal filter bank. *Computers in Biology and Medicine*.

[31] Acharya U. R., Fujita H., Adam M. (2017). Automated characterization and classification of coronary artery disease and myocardial infarction by decomposition of ECG signals: a comparative study. *Information Sciences*.

[32] Kumar M., Pachori R., Acharya U. (2017). Automated diagnosis of myocardial infarction ECG signals using sample entropy in flexible analytic wavelet transform framework. *Entropy*.

[33] Bhaskar N. A. (2015). Performance analysis of support vector machine and neural networks in detection of myocardial infarction. *Procedia Computer Science*.

[34] de Couto G., Ouzounian M., Liu P. P. (2010). Early detection of myocardial dysfunction and heart failure. *Nature Reviews Cardiology*.

[35] Juarez-Orozco L. E., Martinez-Manzanera O., Storti A. E., Knuuti J. (2019). Machine learning in the evaluation of myocardial ischemia through nuclear cardiology. *Current Cardiovascular Imaging Reports*.

[36] Bhoi A. K., Sherpa K. S., Khandelwal B. (2018). Arrhythmia and ischemia classification and clustering using QRS-ST-T (QT) analysis of electrocardiogram. *Cluster Computing*.

[37] Bhoi A. K., Sherpa K. S. (2016). Statistical analysis of QRS-complex to evaluate the QR versus RS interval alteration during ischemia. *Journal of Medical Imaging and Health Informatics*.

[38] Han G., Xu Z. (2016). Electrocardiogram signal denoising based on a new improved wavelet thresholding. *Review of Scientific Instruments*.

[39] Vassilikos V. P., Mantziari L., Dakos G. (2014). QRS analysis using wavelet transformation for the prediction of response to cardiac resynchronization therapy: a prospective pilot study. *Journal of Electrocardiology*.

[40] Jayachandran E. S., Joseph K. P., Acharya U. R. (2010). Analysis of myocardial infarction using discrete wavelet transform. *Journal of Medical Systems*.

[41] Wold S., Esbensen K., Geladi P. (1987). Principal component analysis. *Chemometrics and Intelligent Laboratory Systems*.

[42] He X., Niyogi P. (2003). Locality preserving projections. *Advances in Neural Information Processing Systems*.

[43] Chen T., Guestrin C. Xgboost: a scalable tree boosting system.

[44] Qi Z., Wang B., Tian Y., Zhang P. (2016). When ensemble learning meets deep learning: a new deep support vector machine for classification. *Knowledge-Based Systems*.

[45] Goldberger A. L., Amaral L. A., Glass L. (2000). PhysioBank, PhysioToolkit, and PhysioNet: components of a new research resource for complex physiologic signals. *Circulation*.

[46] Li R., Zhang X., Dai H., Zhou B., Wang Z. (2019). Interpretability analysis of heartbeat classification based on heartbeat activity’s global sequence features and BiLSTM-attention neural network. *IEEE Access*.

[47] Padhy S., Dandapat S. (2017). Third-order tensor based analysis of multilead ECG for classification of myocardial infarction. *Biomedical Signal Processing and Control*.

[48] Liu W., Huang Q., Chang S., Wang H., He J. (2018). Multiple-feature-branch convolutional neural network for myocardial infarction diagnosis using electrocardiogram. *Biomedical Signal Processing and Control*.

